The article "Effects of Combined Spinal Epidural Anesthesia in Orthopaedic Surgery of Elderly Patients" was retracted in 2023. Reasons: signs of a paper mill; compromised peer review; unreliable results or conclusions.

# Effects of Combined Spinal Epidural Anesthesia in Orthopaedic Surgery of Elderly Patients

**DOI:** 10.1155/2022/3523172

**Published:** 2022-10-13

**Authors:** Wei Li, Yingming Fan, Wanghao Chen

**Affiliations:** Department of Anesthesiology, Jingxian Hospital, Jingxian, Xuancheng, Anhui 242500, China

## Abstract

**Objective:**

Combined spinal epidural anesthesia (CSEA) is applied to lower limb orthopaedic surgery in the elderly. This study is aimed at exploring the effect of CSEA in orthopaedic surgery of elderly patients.

**Methods:**

A total of 40 elderly patients with femoral fracture needing hip replacement or femoral head replacement in our hospital from June 2021 to June 2022 were selected as the research objects. The subjects were divided into observation group (*n* = 20) and control group (*n* = 20) by random number table method. The control group was given epidural anesthesia, while the observation group was given CSEA. Hemodynamic indexes (heart rate (HR) and mean arterial pressure (MAP)), visual analogue scale (VAS) pain score changes, anesthetic effects, and postoperative complications were compared between the two groups.

**Results:**

After operation, the observation group had lower HR and MAP values than the control group (*P* < 0.05). The dosage of local anesthetics in the observation group was significantly less than that in the control group (*P* < 0.05). The onset time and improvement time of sensory block in the observation group were significantly faster than those in the control group (*P* < 0.05). The observation group had a lower VAS score than the control group (*P* < 0.05). There was no significant difference in Bromage score or incidence of complications between the two groups (*P* > 0.05).

**Conclusion:**

The use of CSEA has good anesthetic effect. It has the disadvantage of no headache after traditional spinal anesthesia, is not limited by time, and can be used for postoperative analgesia, which is more suitable for the anesthesia of lower limb orthopaedic surgery in the elderly.

## 1. Introduction

In the current aging society of our country, there are more and more elderly surgical cases, and the requirements for surgical anesthesia are becoming higher and higher. As the general physiological function of the elderly is reduced and their tolerance to anesthesia and surgery is poor, the choice of anesthesia for elderly patients undergoing lower limb surgery is a contradictory problem [1, 2]. General anesthesia methods include epidural anesthesia, spinal anesthesia, and combined spinal epidural anesthesia. Lumbar anesthesia interferes with the respiratory and circulatory system. Anesthesia takes effect quickly. Once the anesthesia level fails to meet the requirements, only intravenous general anesthetics can be added to complete the operation, which increases the management difficulty and has time limit. If the operation time is too long, it is difficult to meet the requirements. In addition, postoperative headache may occur during spinal anesthesia, which is the most painful problem for patients after spinal anesthesia, making anesthesiologists and surgeons worried about spinal anesthesia [3, 4]. Epidural anesthesia has the advantages of less interference to the respiratory and circulatory system, less physiological impact, faster postoperative recovery, less complications, etc. [5]. However, it is easy to cause circulatory respiratory depression when applied to the elderly to shorten the onset time, reduce the local anesthetics required for the wide block plane, and strengthen the management at the same time [6]. For example, it is a safe anesthesia method to use small-dose fractional injection; however, there are some problems, such as incomplete epidural anesthesia, especially adhesion in the epidural space caused by multiple epidural anesthesia, and the diffusion of local anesthetics is blocked. Epidural catheter entering into intervertebral foramen resulted in limited block range; and there may be unilateral anesthesia. The circulatory and respiratory disturbance caused by intravenous general anesthetics during incomplete block increases the risk of anesthesia and the difficulty of management [7].

The article "Effects of Combined Spinal Epidural Anesthesia in Orthopaedic Surgery of Elderly Patients" was retracted in 2023. Reasons: signs of a paper mill; compromised peer review; unreliable results or conclusions.

For most orthopaedic operations, such as total hip arthroplasty or knee arthroplasty, regional anesthesia is better than general anesthesia. Most regional block, such as spinal anesthesia and epidural anesthesia, can obtain good anesthetic effect during the operation, facilitate the operation, and control the pain well after the operation. Combined spinal epidural anesthesia (CSEA) is a combination of subarachnoid block and epidural catheter indwelling [8, 9]. Combined spinal epidural anesthesia has the advantages of rapid onset and good analgesic and muscle relaxation effect and is widely used in orthopaedic surgery [10]. In addition, it has been reported that CSEA is also applied for caesarean section and breast surgery [11, 12]. Elderly patients have many basic diseases and high perioperative anesthesia risk. Therefore, choosing an ideal anesthesia scheme is of great significance to stabilize intraoperative hemodynamics and reduce anesthesia risk [13]. The purpose of this study was to explore the effect of combined spinal epidural anesthesia in elderly patients undergoing orthopaedic surgery through clinical trials.

## 2. Materials and Methods

### 2.1. Clinical Data

A total of 40 elderly patients with femoral fracture who planned to undergo hip replacement or femoral head replacement in our hospital from June 2021 to June 2022 were selected as the research objects. This study was approved by the Ethics Committee of our hospital. The subjects were divided into observation group and control group by random number table method, with 20 cases in each group. In the observation group, there were 11 males and 9 females; the average age was 74.32 ± 8.27 years. In the control group, there were 10 males and 10 females; the average age was 75.16 ± 8.33 years. There was no significant difference between the two groups (*P* > 0.05).

The article "Effects of Combined Spinal Epidural Anesthesia in Orthopaedic Surgery of Elderly Patients" was retracted in 2023. Reasons: signs of a paper mill; compromised peer review; unreliable results or conclusions.

Inclusion criteria are as follows: patients who underwent elective surgery; age > 60; American Society of anesthesiologists (ASA) grade I or II; there were no serious pathological changes of important organs before operation; the operation time was less than 2 hours; and those who agree to participate in the study and sign the informed consent form.

Exclusion criteria as follows: long-term use of analgesic and sedative drugs; preoperative blood glucose and blood pressure were not effectively controlled; severe coagulation dysfunction; the skin at the puncture site is broken; severe deformity of spine; contraindication of intraspinal anesthesia; and history of acute and chronic pain.

### 2.2. Methods

*Epidural anesthesia*: the control group used epidural anesthesia: (1) intramuscular injection of atropine 0.5 mg and diazepam 10 mg 30 min before operation. 3~4 ml of 1.5% lidocaine was given for local anesthesia, and 3~6 ml was added after ensuring that there was no abnormality. (2) Oxygen inhalation with mask and ECG monitoring. (3) If the intraoperative blood pressure drops significantly, ephedrine 5-10 mg should be given intravenously until it rises. Patients with ventricular premature beats should be given lidocaine 50~100 mg intravenously until it disappears.

*Combined spinal epidural block anesthesia*: the observation group used combined spinal epidural block anesthesia. After entering the operating room, open the venous channel to quickly input Hess for routine monitoring of ECG, blood pressure, oxygen saturation, and oxygen inhalation, and then, perform right internal jugular vein or right subclavian vein puncture for central venous pressure (CVP) measurement to evaluate intraoperative bleeding and infusion, which can be used for intraoperative rapid infusion and blood transfusion. Take the patient with slightly higher head and lower foot to lie on the side and select the lumbar 2~3 space for puncture. After reaching the epidural space, perform subarachnoid puncture with 25G lumbar puncture needle. After cerebrospinal fluid outflow is seen, give 0.75% bupivacaine 1 ml~1.3 ml plus 25% glucose 0.2 ml~0.3 ml mixed solution and place a catheter in the epidural space. Monitor the anesthesia level at any time and adjust the anesthesia level through body position change to control the anesthesia level not to exceed T8. The operation can be performed after the anesthesia level is stable. In the epidural group, 0.75% ropivacaine was used. In both groups, the analgesic pump was used. The analgesic drug was ropivacaine 150 mg, morphine 4 mg, and normal saline to 100 ml.

The article "Effects of Combined Spinal Epidural Anesthesia in Orthopaedic Surgery of Elderly Patients" was retracted in 2023. Reasons: signs of a paper mill; compromised peer review; unreliable results or conclusions.

### 2.3. Observation Indicators

1. Record HR and MAP before anesthesia (T0), before operation (T1), 30 min after operation (T2), immediately after operation (T3), and 15 min after operation (T4)
2. VAS pain score changes before and after anesthesia in the two groups. The core range was 0-10: severe: 7~10 points; moderate: 4~6 points; mild: 1~3 points; and painless: 0 points
3. The anesthetic effects of the two groups were compared. Lower limb motor nerve block was measured by modified Bromage method (grade 0: no motor nerve block; grade 1: unable to lift the leg; grade 2: unable to bend the knee; and grade 3: unable to bend the ankle)
4. The occurrence of postoperative complications in the two groups, such as shivering, decreased blood pressure, slower heart rate, nausea, vomiting, and postoperative headache
5. Anesthesia of the two groups. The local anesthetic dosage, onset time of sensory block, block plane, block completion time, pain recovery time, auxiliary drugs, blood loss, and infusion volume were compared between the two groups

### 2.4. Statistical Analysis

The measurement data are expressed as mean ± standard deviation (*x* ± *s*) and *t*-test or *χ*^2^. Carry out statistical analysis. *P* < 0.05 was considered as statistically significant.

## 3. Results

### 3.1. Comparison of Anesthesia between the Two Groups

The dosage of local anesthetics, onset time of sensory block, block completion time, and pain recovery room in the observation group were significantly less than those in the control group (*P* < 0.05), as shown in Table 1.

### 3.2. Comparison of HR and MAP between the Two Groups during Operation

HR and MAP at T2 and T3 time points in the control group were higher than those at T0, T1, and T4time points (*P* < 0.05). HR at T2, T3, and T4 in the observation group was lower than that at T0 and T1 (*P* < 0.05). The HR of patients in the observation group at T2, T3, and T4 time points was lower than that in the control group (*P* < 0.05). The MAP of patients in the observation group at T2, T3, and T4 time points was lower than that in the control group (*P* < 0.05). There were no significant difference of HR and MAP at T0 and T1 time points between the two groups (*P* > 0.05), as seen in Figure 1.

The article "Effects of Combined Spinal Epidural Anesthesia in Orthopaedic Surgery of Elderly Patients" was retracted in 2023. Reasons: signs of a paper mill; compromised peer review; unreliable results or conclusions.

### 3.3. Comparison of Anesthetic Effects between the Two Groups

As shown in Figure 2, there was no significance of Bromage score between the two groups (*P* > 0.05).

### 3.4. Comparison of VAS Pain Scores between the Two Groups before and after Operation

There was no significant change in the preoperative VAS pain score of the two groups (*P* > 0.05). The VAS pain score at the time of awakening after operation was increased significantly and showed a downward trend 24 hours after operation. The VAS pain score in the control group was higher than that in the observation group, the difference was statistically significant (*P* < 0.05), as seen in Figure 3.

### 3.5. Comparison of Postoperative Complications between the Two Groups

The incidence of complications including chills, low blood pressure, slowed heart rate, nausea and vomiting, and headaches in the observation group was lower than that in the control group, but the difference was not statistically significant (*P* > 0.05), as seen in Figure 4.

## 4. Discussion and Conclusion

CSEA absorbs the advantages of epidural anesthesia and spinal anesthesia. As long as the anesthesia level is controlled below T8, it has little interference on circulation and respiration, and the anesthesia effect is good. At the same time, the operation is basically completed within 2 h. Generally, the operation can be completed without adding local anesthetics, so as to avoid incomplete epidural anesthesia block. At the same time, the local anesthetics dose required is small, which also reduces the occurrence of toxic and side effects of local anesthetics, and the postoperative recovery is fast, with less complications [14]. Because the CSEA lumbar puncture needle is thinner than the traditional lumbar anesthesia needle, there are no headache complications in the postoperative follow-up. This is mainly because the 25 g pen point SA needle is used to puncture the dura mater in a separate way, with relatively few dots and less cerebrospinal fluid outflow, and CSEA is not limited by time. The anesthesia time can be extended arbitrarily according to the needs of the operation. PCEA analgesia or treatment is feasible after the operation.

This study showed that both groups of anesthesia planes could meet the requirements of surgery and had little impact on the body. Combined spinal epidural anesthesia not only has the advantages of fast onset, muscle relaxation, and perfect analgesia but also can effectively adjust the anesthesia plane to prevent the high anesthesia plane [15]. Small-dose bupivacaine given in combined spinal epidural anesthesia can provide anesthesia plane in a short time and reduce the degree of interference to respiratory and circulatory system, and small dose can significantly reduce intravascular local anesthetic drugs and reduce the risk of local anesthetic drug poisoning [15, 16]. Meanwhile, the results of this study showed that the VAS pain score, hemodynamic index changes, and anesthesia index of the observation group were better than those of the control group, which was mainly related to the fact that intraspinal anesthesia can lead to significant preganglionic block of the sympathetic nerve in the block area, dilation of blood vessels, insufficient blood volume, and cardiac output [17]. In addition, elderly patients have a certain degree of autonomic and peripheral nerve degenerative changes. When the body is under anesthesia, the catecholamine level can be reduced during anesthesia. In addition, their body position changes after anesthesia, resulting in large changes in hemodynamic indicators [18]. The index parameters of the observation group were all within 20% of the basic value, indicating that it had little interference with the circulatory system.

The article "Effects of Combined Spinal Epidural Anesthesia in Orthopaedic Surgery of Elderly Patients" was retracted in 2023. Reasons: signs of a paper mill; compromised peer review; unreliable results or conclusions.

However, the number of patients in this study was relatively small. Future validation studies are warranted, preferably in a prospective setting.

To sum up, CSEA has the advantages of good anesthetic effect when it is used in lower limb orthopaedic surgery for the elderly. When the anesthesia level is controlled below T8, it has the advantages of little impact on the circulatory and respiratory system, rapid postoperative recovery, less complications, and no headache after traditional spinal anesthesia. In addition, epidural anesthesia is not limited by time and has the advantages of feasible postoperative analgesia, so it is a more suitable anesthesia method for lower limb orthopaedic surgery in the elderly.

## Figures and Tables

**Figure 1:** Comparison of HR and MAP between the two groups during operation. Note: compared with the control group, ^∗^*P* < 0.05.

**Figure 2:** Comparison of anesthetic effects between the two groups.

**Figure 3:** Comparison of VAS pain scores between the two groups before and after operation. Note: compared with the control group, ^∗^*P* < 0.05.

**Figure 4:** Comparison of postoperative complications between the two groups.

**Table 1:** Comparison of anesthesia between the two groups.

Groups	*N*	Local anesthetic dosage (mg)	Onset time of sensory block (s)	Blocking plane	Block completion time (min)	Pain recovery room (min)
Control group	20	85.0 ± 21.5	246.0 ± 58.0	T_10_ (T_08~11_)	20.0 ± 5.5	165.0 ± 29.6
Observation group	20	8.0 ± 1.6^∗^	42.0 ± 11.0^∗^	T_10_ (T_08~11_)	9.0 ± 4.8^∗^	126.0 ± 24.7^∗^

Note: compared with the control group, ^∗^*P* < 0.05.

The article "Effects of Combined Spinal Epidural Anesthesia in Orthopaedic Surgery of Elderly Patients" was retracted in 2023. Reasons: signs of a paper mill; compromised peer review; unreliable results or conclusions.

## Data Availability

Data generated in this study are available from the corresponding author upon reasonable request.
